The article "How Residents' Attitudes to Tourists and Tourism Affect Their Pro-tourism Behaviours: The Moderating Role of Chinese Traditionality" was retracted in 2025. Reasons: unreliable results or conclusions; a conflict of interest; concerns about the peer review; concerns about the citations.

# How Residents' Attitudes to Tourists and Tourism Affect Their Pro-tourism Behaviours: The Moderating Role of Chinese Traditionality

**DOI:** 10.3389/fpsyg.2021.792324

**Published:** 2022-01-21

**Authors:** Ke Shen, Jian Yang, Chuan Geng

**Affiliations:** ^1^School of Tourism, Huangshan University, Huangshan, China; ^2^School of Journalism and Communication, Guangzhou University, Guangzhou, China; ^3^School of Economics and Management, Hainan Normal University, Haikou, China

**Keywords:** host-tourist interaction, place image, attitudes to tourism, attitudes to tourist, Chinese traditionality, pro-tourism behaviours

## Abstract

Although sufficient attention has been paid to residents' attitudes to tourism in previous studies, few studies have used residents' attitudes to tourists and tourism simultaneously to explain their support for tourism. This study fills this gap by examining the effect of place image and host–tourist interactions on residents' attitudes to tourists and tourism, respectively, and their consequent reactions by considering the moderating effect of Chinese traditionality. The proposed model is tested using data from 357 residents living in Huangshan, a fifth-tier city in China. Results demonstrate that attitudes to tourism and host-tourists interaction positively affect their pro-tourism behaviours. Moreover, attitudes to tourism mediate place the image's, host–tourists interaction's and attitudes to tourists' respective relationships with pro-tourism behaviours. Furthermore, the higher the Chinese traditionality of residents, the stronger the influence of their attitudes to tourism on pro-tourism behaviours. However, the relationship of place image and attitudes of residents towards tourists with pro-tourism behaviours are not supported. Findings offer critical implications for planners, practitioners and interested researchers.

## Introduction

Rural tourism is a type of tourism that began and thoroughly developed in Europe as a result of industrialisation and urbanisation (Wang et al., 2013; Cuadrado-Ciuraneta et al., 2017). Rural tourism has greatly contributed to economic development, especially in rural areas. Therefore, governments worldwide have adopted various measures to promote rural tourism. For instance, the Austrian government provides preferential loans or even subsidies to support rural tourism businesses. Education has played an extremely important role in the development of rural tourism beyond financial promotion in France (Pakurár and Olah, 2008). A new policy, namely the “Pays d' Accueil,” was even introduced by the French government to attract tourists to rural areas in 1976 (Keane, 1992). In recent years, the Chinese government has strengthened its support for rural economic growth, established the Rural Revitalization Bureau and viewed tourism development as one of the most essential ways to boost rural economic development (Liu et al., 2020). However, rural tourism is bound to bring effects to tourist destinations, such as reducing local environmental performance (Usman et al., 2020; Musa et al., 2021) and even to local residents themselves (Wang et al., 2021). Consequently, various tourist attractions have recently experienced an increase in open hostility towards tourists as part of residents' efforts to combat tourism development (Zaman and Aktan, 2021). Thus, investigating residents' opinions about tourism is urgent and beneficial.

The article "How Residents' Attitudes to Tourists and Tourism Affect Their Pro-tourism Behaviours: The Moderating Role of Chinese Traditionality" was retracted in 2025. Reasons: unreliable results or conclusions; a conflict of interest; concerns about the peer review; concerns about the citations.

Local residents' support for tourism has been recognised in the literature because it determines the success and sustainability of tourist destinations (Gursoy and Rutherford, 2004; Ward and Berno, 2011). Ribeiro et al. (2017) have even advocated that it is an essential prerequisite for the sustainability of any tourist destination. Thus, many types of research have been conducted to explore new predictors of residents' support for tourism. However, the majority of studies in this field are focused primarily on residents' attitudes to tourism (ATT). None of these studies have considered residents' attitudes to tourists (ATTT) (Woosnam, 2011; Monterrubio, 2016), and few studies have identified why and how residents form and develop their attitudes (Sharpley, 2014). Even fewer studies have investigated residents' ATT and ATTT simultaneously to explain their support for tourism. One exception is a study by Martín et al. (2018), which includes attitudes to tourism in general and tourists in particular to explain why residents hold a high level of support for tourism.

Research also suggests that understanding residents' place image (PI) is important to understand their attitudes and behaviours (Stylidis et al., 2014). However, the influence of PI on residents' support for tourism has been under-examined (Stylidis, 2016). Despite host–tourist interactions (HTI) having been identified as a critical issue in the tourism industry (Ward and Berno, 2011), studies on HTI are mainly focused on the effect of such interactions on tourists' experiences (Luo et al., 2015; Chen et al., 2018). Consequently, the effects of HTI on residents' support for tourism is under-researched (Fan et al., 2017b; Eusébio et al., 2018). In addition, a large body of research suggests that many factors, such as personality traits (Kim et al., 2021), gender (Casado-Díaz et al., 2020) and green marketing (Liao et al., 2020), motivation (Kim et al., 2017) moderate the links between attitudes and intention. However, research examining the cultural boundaries of the utility of attitudes on intention is scarce. Furthermore, “cultural values are also influential in altering the relationship between antecedents and silence behaviour” (Wan et al., 2021) and several variations in attitudes and behaviour patterns occur between groups with high and low levels of Chinese traditionality (CT) (Wang et al., 2020). From a resident perspective, some scholars have begun to explore the relationship between PI, HTI, attitudes and pro-tourism behaviours (PBI) (Tosun et al., 2020; Zaman and Aktan, 2021; Tse and Tung, 2022), but these efforts are far from sufficient. Therefore, the research gap necessitates expanding the literature in this field to understand why residents support tourism in their communities and how the influencing factors affect each other. To be specific, the scientific discourse should increase its emphasis on deeper examinations of residents' HTI, PI, CT and attitudes to achieve sustainable tourism development (Wang and Zhang, 2020; Xiong et al., 2021; Zaman and Aktan, 2021).

The article "How Residents' Attitudes to Tourists and Tourism Affect Their Pro-tourism Behaviours: The Moderating Role of Chinese Traditionality" was retracted in 2025. Reasons: unreliable results or conclusions; a conflict of interest; concerns about the peer review; concerns about the citations.

Given these considerations, this study aims to introduce HTI and PI within current research on residents' attitudes and behaviours, examine the effect of HTI and PI on residents' ATT and ATTT as well as their support for tourism by considering the moderating effect of CT and assess the relationship between both types of attitudes. Thus, the findings of this study would shed light on the planning and management practises of places as tourist attractions.

The remainder of this study is organised as follows. In section Literature Review, a review of literature on every variable is introduced, and the hypotheses among the variables are developed. In section Methodology, the methodology is explained, and the profiles of the informants are summarised. In Section Results, the findings are reported. In section Discussion and Conclusions, the findings are discussed and concluded. In section Theoretical and Practical Implications, theoretical and managerial implications are provided. In section Limitations and Future Research, limitations and directions for future studies are given.

## Literature Review

### Residents' Pro-tourism Behaviours

Different from some previous studies that regard the concept of residents' support for tourism in terms of attitudes (Nunkoo and So, 2016), this study regards it as residents' PBI, which refers to how much effort residents would exert to support tourism development. In consideration of the importance of residents' support for tourism, many studies have explored the antecedents of such support, including tourism impact (Papastathopoulos et al., 2019), personal benefit (Gursoy et al., 2019), ATT (Ribeiro et al., 2017), state of local economy (Garau-Vadell et al., 2019), emotion (Maruyama et al., 2019) and place attachment (Kang, 2019). Recently, some new variables have been considered to explain residents' support. These variables include ambivalence (Chen et al., 2019), tourism ethnocentrism (Kock et al., 2019), travel use history (Woosnam et al., 2018), collaboration (Phuc and Nguyen, 2020), cultural intelligence (Zaman and Aktan, 2021) and perceived risk (Joo et al., 2021). A review of the literature suggests that most prior studies are atheoretical (Nunkoo et al., 2013). However, to a certain extent, the atheoretical studies made generalising results difficult. Scholars have therefore tried to conduct research based on a variety of theories, the most widely used of which are social exchange theory followed by social representations theory (Bimonte and Punzo, 2016; Hadinejad et al., 2019).

The article "How Residents' Attitudes to Tourists and Tourism Affect Their Pro-tourism Behaviours: The Moderating Role of Chinese Traditionality" was retracted in 2025. Reasons: unreliable results or conclusions; a conflict of interest; concerns about the peer review; concerns about the citations.

To sum up, two research streams focus on exploring the antecedents of residents' support for tourism, namely, economic and non-economic (Hu et al., 2019). The economic stream mainly consists of factors such as personal benefits, assessments of the economic effects of tourism and tradeoffs between the positive and tourism impacts. The non-economic stream mainly consists of factors such as residents' empowerment, sociodemographic factors and length of residence.

### Residents' Attitudes to Tourism and Tourists

Attitudes typically encompass three dimensions: cognitive, affective and behavioural (Carmichael, 2000). However, the study of attitudes has mainly focused on the behavioural dimension, and the other two dimensions of residents' attitudes, namely, cognitive and affective, have been almost ignored (Monterrubio, 2016). Thus, in this study, residents' attitudes are focused on those two dimensions, which aim to distinguish themselves from residents' PBI. Previous studies on residents' attitudes are mainly exploratory and descriptive. Why and how such attitudes develop and are predicted are questions that require further examination (Monterrubio, 2016). Eusébio et al. (2018) has drawn a similar conclusion. The literature thus far has substantiated that residents' PBI is mostly affected by ATT (Nunkoo and Gursoy, 2012). In a study of 418 residents from the Cape Verde Islands, Ribeiro et al. (2017) found that their ATT effects significantly influenced their PBI. In Zhuhai City (China), Wang and Xu (2015) found that residents' ATT significantly affected their support for tourism. With a sample of 300 residents in Mauritius, Nunkoo and Gursoy (2012) found that their attitudes to positive and negative tourism impacts significantly affected their support for island tourism. Using a sample of 766 residents from three destination areas, Kwon and Vogt (2010) found that residents' attitudes to place marketing were positively related to place marketing activities in all three destination areas. Thus, the following hypothesis is proposed:

H1: Residents' ATT positively influence their PBI.

The article "How Residents' Attitudes to Tourists and Tourism Affect Their Pro-tourism Behaviours: The Moderating Role of Chinese Traditionality" was retracted in 2025. Reasons: unreliable results or conclusions; a conflict of interest; concerns about the peer review; concerns about the citations.

Given that ATTT concerns host–guest interaction, destination image, tourists' experience and even sustainable tourism development, research on residents' ATTT would be of major importance (Tse and Tung, 2022). However, the majority of previous studies are primarily focused on residents' ATT (Woosnam, 2011; Monterrubio, 2016). To the best of our knowledge, few studies have been undertaken on residents' ATTT (Palmer et al., 2013; Monterrubio, 2016; Chen et al., 2018; Egresi and Kara, 2018; Joo et al., 2018; Martín et al., 2018), and no research has simultaneously explored the relationship between residents' ATT and ATTT. With 39 semi-structured interviews with Hong Kong residents, Chen et al. (2018) found that residents' unfavourable attitudes to Mainland Chinese tourists exceeded neutral or positive ATT. Following the “perceptions–attitudes–behaviours” sequence, Martín et al. (2018) found that residents' perception of tourism impacts was the main factor affecting their ATT and ATTT, in turn influencing residents' behavioural support for tourism in host communities. With a sample of 583 residents from Istanbul, Turkey, Egresi and Kara (2018) found that local communities were supportive of tourists, although different demographics, cultural backgrounds and the number of tourists would also change their attitudes. In 27 in-depth interviews with Cancun residents (Mexico), Monterrubio (2016) found that realistic threats and intergroup anxiety were the main predictors of residents' pre-judicial ATTT. However, none of the above studies explored the consequences of residents' ATTT on other variables, not to mention the relationship between their ATT and ATTT.

In a study by Martín et al. (2018), residents' ATT and ATTT were found to be related to residents' behaviours supporting tourism in their communities. In an investigation of 307 Welsh residents, Palmer et al. (2013) confirmed the direct positive association between residents' affective ATTT and residents' propensity to engage in positive advocacy to support inward tourism. Moreover, Woosnam (2012) argued that residents' feelings about tourists are an essential prerequisite for residents' PBI. Thus, the following hypothesis is proposed:

H2: Residents' ATTT positively influence their PBI.

The article "How Residents' Attitudes to Tourists and Tourism Affect Their Pro-tourism Behaviours: The Moderating Role of Chinese Traditionality" was retracted in 2025. Reasons: unreliable results or conclusions; a conflict of interest; concerns about the peer review; concerns about the citations.

Until recently, researchers began to explore ATT through ATTT (Shen et al., 2017). An emotional solidarity scale to measure residents' ATTT was developed in previous studies (Woosnam, 2011, 2012). Woosnam and Aleshinloye (2018) reported that emotional solidarity is subject to the degree of one's identification with another. Woosnam (2012) found that all three sub-dimensions of emotional solidarity significantly affected residents' ATT. Hasani et al. (2016) found that residents' level of welcoming nature to tourists is related to their ATT. Woosnam (2012) also reported that residents' ATTT may affect their ATT. Such a research direction remains insufficient in existing research. Thus, we propose the following hypotheses:

H3: Residents' ATTT positively influence their ATT.
H3a: Residents' ATT positively mediate the relationship between their ATTT and PBI.

### Host–Tourist Interaction

HTI refers to personal encounters between tourists and hosts (Yvette and Turner, 2003). As a critical component of tourism experience and a complex construct in the field of travel and tourism, HTI has been conceptualised in different ways (Eusébio et al., 2018). No agreement has been reached in terms of how to measure HTI and what the consequences of HTI are (Eusébio et al., 2016, 2018). The frequency of and satisfaction with an interaction are more commonly used to measure HTI (Eusébio et al., 2018). Joo et al. (2018) used frequency and the nature of interactions to measure HTI and explored their effect on social distance and emotional solidarity. Luo et al. (2015) examined the influence of HTI, encompassing two dimensions, namely, quality and quantity, of interactions on residents' perceptions of backpackers and evaluations of backpackers' effects. Fan et al. (2017a) also used the same measure to understand HTI. Kirillova et al. (2015) used frequency and quality (content) to evaluate HTI and found that quality was the most influential factor in changing intercultural sensitivity.

Although HTI is vital to understanding the influence of tourism on local communities in tourist destinations (Zhang et al., 2017), most previous studies have focused mainly on the influence of HTI on visitors' satisfaction, intention to return and hosts' satisfaction. Most of these studies were conducted in developed countries (Eusébio et al., 2016). Given the different reactions to tourism in developed and developing countries (Sirakaya et al., 2002), whether the strength of HTI on residents' attitudes and consequent reactions in developing countries is the same as that in developed countries needs to be confirmed.

Fan et al. (2017a) argue that tourists and hosts are essential in HTI, making HTI bidirectional, namely, HTI can be rewarding experiences that develop cultural understanding for tourists and provide positive influences on the social and cultural lives of residents (Su et al., 2016). On the one hand, some researchers have examined HTI from tourists' perspectives and the influence of HTI on tourists' satisfaction with their stay and destination experience (Pizam et al., 2000; Su et al., 2016; Fan et al., 2019). Other researchers have examined such issues as the effect of HTI on tourists' perceived cultural distance (Fan et al., 2017b), their willingness to pay (Bimonte and Punzo, 2016) and their intercultural sensitivity (Kirillova et al., 2015). On the other hand, some studies on HTI have been conducted from the perspectives of residents to examine various effects of HTI on factors such as residents' ATT (Eusébio et al., 2018), emotional solidarity and social distance (Joo et al., 2018), tourism impacts (Carneiro et al., 2018) and perception of tourists. Some studies on HTI have also been undertaken from residents' and tourists' perspectives (Kastenholz et al., 2013; Bimonte and Punzo, 2016; Su et al., 2016; Zhang et al., 2017).

The article "How Residents' Attitudes to Tourists and Tourism Affect Their Pro-tourism Behaviours: The Moderating Role of Chinese Traditionality" was retracted in 2025. Reasons: unreliable results or conclusions; a conflict of interest; concerns about the peer review; concerns about the citations.

Positive intergroup contact can reduce pre-judice and anxiety, and pre-judice can reduce contact (Binder et al., 2009). In the context of tourism, some predictors of positive attitudes change due to contact and HTI may cause positive ATTT (Joo et al., 2018). Sharpley (2018) also argued that interactions may influence hosts' attitudes, opinions and, ultimately, lifestyles. Based on contact hypothesis and integrated threat theory, Ward and Berno (2011) found that more frequent and satisfying interactions (contact) with tourists cause positive ATTT. Through research in Lijiang, China, Luo et al. (2015) found that the quality of HTI between hosts and backpackers affected local residents' perceptions of tourists (backpackers). Also, Eusébio et al. (2018) found that HTI is related to residents' perceived positive effects and their ATT. More recently, Xiong et al. (2021) found that HTI quality was positively related to their attitudes towards tourism development. Thus, we put forward the following hypotheses for testing:

H4: Residents' HTI positively influence their ATT.
H5: Residents' HTI positively influence their ATTT.
H6: Residents' HTI positively influence their PBI.
H6a: Residents' ATT positively mediate the relationship between their HTI and PBI.

### Residents' Place Image

PI is defined as the combination of beliefs, thoughts and expressions people have about a place (Rein et al., 1993). The influence of PI on an individual's behaviour has been examined in many disciplines. However, previous tourism studies have exposed a lack of studies regarding local residents' image of the place where they live and work (Stylidis, 2018; Shen et al., 2019). Most previous studies have focused mainly on tourists' PI, especially its influence on tourists' revisit intention (Stylos et al., 2017), intention to recommend (Qu et al., 2011), satisfaction (Lee, 2009), destination attachment (Zhang et al., 2019), loyalty (Hungenberg et al., 2019) and emotion (Xu et al., 2019). Only a few studies have concentrated on residents' perspectives (Stylidis et al., 2014; Stylidis, 2018). With a sample of 481 residents of Kavala, Greece, Stylidis et al. (2018) argued that three distinct resident groups with different PI perceptions exhibit dissimilar ATT. In an investigation of 368 residents of Eilat, Stylidis (2018) found that residents with the most favourable image of Eilat tend to support tourism development much more than do the residents with the least favourable image of Eilat. In Colorado, Kang (2019) found that the state image and cannabis image of local residents are both related to their support for marijuana tourism. In a study by Stylidis et al. (2014), residents' PI was found to be important in shaping their support for tourism development. Similarly, Chang et al. (2020) found that that residents' PI was positively related to their support for sports tourism development. To the best of our knowledge, no study has tested the direct influence of residents' PI on their ATTT. Our study tests this relationship using PLS-SEM, which is especially suitable for prediction and exploratory research (Hair et al., 2019). Thus, residents' PI might have a significant influence on their ATTT. Accordingly:

H7: Residents' PI positively influences their ATTT.
H8: Residents' PI positively influences their ATT.
H9: Residents' PI positively influences their PBI.
H9a: Residents' ATT positively mediate the relationship between their PI and PBI.

The article "How Residents' Attitudes to Tourists and Tourism Affect Their Pro-tourism Behaviours: The Moderating Role of Chinese Traditionality" was retracted in 2025. Reasons: unreliable results or conclusions; a conflict of interest; concerns about the peer review; concerns about the citations.

### Chinese Traditionality

Traditionality was defined as a commitment to, respect for and acceptance of customs and norms of a traditional society (Schwartz, 1992). Rooted in Confucian ideology, CT was originally developed in the 1980s and defined as “the typical pattern of more or less related motivational, evaluative, attitudinal and temperamental traits” (Yang, 2003). Individuals with high levels of CT are more inclined to display the following five characteristics: submission to authority, filial piety and ancestor worship, conservatism and endurance, fatalism and defensiveness and male dominance (Yang et al., 1989). Submission to authority is the only characteristic correlating positively with the other four (Farh et al., 2007). Thus, CT is thought to represent the cultural value of one's submission to authority in this study, consistent with some previous studies (Farh et al., 1997; Wang and Zhang, 2020).

Farh et al. (1997) introduced the concept of CT from social psychology into organisational behaviour and argued that individuals with varying levels of CT exhibited a wide range of attitudes and behaviours, as confirmed in subsequent studies (Wang and Zhang, 2020; Yang et al., 2020; Xu et al., 2021). However, most previous studies on CT are mainly concentrated in human resource management (Wang et al., 2020; Wan et al., 2021; Xu et al., 2021). CT research in travel and tourism remains scarce.

Azjen (1980) suggests that the effect of individual attitudes on their intention formation may be determined by their value priorities. Wang et al. (2020) argued that CT is an important value influencing factor that constrains modern Chinese behaviour. Specifically, several variations in attitudes and behaviour patterns were found between the high and low CT groups (Wang et al., 2020). Moreover, cultural values “are also influential in altering the relationship between antecedents and silence behaviour” (Wan et al., 2021). This postulation is also supported by empirical evidence. Based on a survey of 370 Chinese Singaporean women, Koubaa et al. (2011) found that CT moderates the relationship between their attitudes towards skin smoothness and skin fairness and willingness to buy cosmetics. Thus, we propose the following hypotheses:

H10: Residents' CT moderates the relationship between their ATT and PBI.
H11: Residents' CT moderates the relationship between their ATTT and PBI.

All hypothesised relationships are demonstrated in Figure 1.

**Figure 1:** Research model with relevant hypotheses.

## Methodology

### Research Instrument

This quantitative study used questionnaires to gather data. We adopted a measurement with four dimensions: physical appearance (PHA), community services (CS), social environment (SE) and entertainment services (ES) to evaluate PI (Stylidis et al., 2014, 2016; Stylidis, 2016). A single item of CS was deleted due to its low factor loading. HTI was assessed with three items adapted from Eusébio et al. (2018). We adapted four items from Palmer et al. (2013) and Martín et al. (2018) to evaluate ATTT. To assess ATT, four items were adapted from Martín et al. (2018). CT was evaluated with five items adapted from Wang and Zhang (2020). Given the similarity between participants and behaviours, the four items from Ribeiro et al. (2017) were used to evaluate PBI. A single item of this variable was deleted due to its unsatisfactory loading value.

We used back-translation to ensure that Chinese questionnaires correctly reflected the meaning of the original English version. A seven-point Likert-type scale was used to assess all measurable items from 1 (strongly disagree) to 7 (strongly agree). The whole questionnaire consisted of two parts. Part 1 comprised 32 items for the 5 variables in this study, and Part 2 comprised 6 questions related to the socio-demographic profile of the participants.

The article "How Residents' Attitudes to Tourists and Tourism Affect Their Pro-tourism Behaviours: The Moderating Role of Chinese Traditionality" was retracted in 2025. Reasons: unreliable results or conclusions; a conflict of interest; concerns about the peer review; concerns about the citations.

### Study Area

Huangshan City is located in the southern part of Anhui Province and is an important tourist city in China. The Huangshan Scenic Area within its territory is a UNESCO World Heritage Site. In 2019, Huangshan City received 74,022,100 tourists, an increase of 14.1% over the previous year, and the total tourism revenue was CNY 65.945 billion, an increase of 15.1%. Tourism income accounts for approximately 40% of the total income of the national economy. Tourism has become an important pillar industry of Huangshan, and Huangshan has become an important tourist destination in China. Huangshan is also working to develop itself as an excellent world tourist destination^1^.

### Sampling and Data Collection

This study selects the surrounding communities of Huangshan Scenic Area for investigation. The area comprises 19 communities, all of which have different levels of tourism development. Owing to the different educational levels of community residents, to facilitate communication and improve communication efficiency between them and the researchers, we invited community staff to participate. In this study, 20 questionnaires were distributed in each community from July 6 to August 1, 2021. Participants were given tokens to encourage participation and thank them for their time spent on the survey. A total of 380 questionnaires were distributed, 380 were returned, and 357 valid questionnaires were collected. The profile of the 357 informants is summarised in Table 1.

**Table 1:** Socio-demographic information of respondents.

**Characteristics**	***N* (357)**	**% (100)**
**Gender**		
Male	163	45.7%
Female	194	54.3%
**Marital status**		
Single	105	29.4%
Married	251	70.3%
Others	1	0.3%
**Age**		
18–25	78	21.8%
26–35	148	41.5%
36–45	75	21.0%
≥46	56	15.6%
**Education**		
Middle school or less	69	19.3%
Junior college	94	26.3%
Undergraduate	163	45.7%
Post-graduate or higher	31	8.7%
**Job**		
Government agent	68	19.0%
Self-employed or Freelancer	78	21.9%
Student	51	14.3%
Office worker	160	44.8%
**Income**		
≤ ¥4,000	75	21.0%
¥4,001–6,000	100	28.0%
¥6,001–8,000	67	18.8%
¥8,001–10,000	71	19.9%
≥¥10,001	44	12.3%

## Results

### Measurement Model

PLS-SEM using SmartPLS version 3.2.8 and SPSS version 25 was chosen to analyse the data because PLS-SEM is especially useful for prediction and exploratory research (Hair et al., 2019). This study follows a two-step procedure comprising the measurement and structural models (Hair et al., 2021). In Table 2, all factor loadings exceed 0.708 suggested by Hair et al. (2019). Cronbach's α (0.881–0.941) and composite reliability (CR) (0.913–0.957) all exceed the recommended levels as suggested by Hair et al. (2019). Thus, satisfactory reliability of the measurement model was established. Average variance extracted (AVE) (≥0.5 as a threshold) is usually chosen to check convergent validity (Hair et al., 2019). In this study, AVE values (0.588–0.881) of each variable all exceed the suggested threshold of 0.5. Thus, the convergent validity is satisfactory.

The article "How Residents' Attitudes to Tourists and Tourism Affect Their Pro-tourism Behaviours: The Moderating Role of Chinese Traditionality" was retracted in 2025. Reasons: unreliable results or conclusions; a conflict of interest; concerns about the peer review; concerns about the citations.

**Table 2:** Results of confirmatory factor analysis.

**Items**	**Factor loading**	**Cronbach's α**	**CR**	**AVE**
**Attitudes to tourism**		0.919	0.943	0.805
ATT1	0.905			
ATT2	0.893			
ATT3	0.915			
ATT4	0.876			
**Attitudes to tourists**		0.937	0.955	0.840
ATTT1	0.936			
ATTT2	0.920			
ATTT3	0.902			
ATTT4	0.908			
**Host-tourist interaction**		0.930	0.956	0.878
HTI1	0.931			
HTI2	0.969			
HTI3	0.910			
**Community services**		0.933	0.957	0.881
CS1	0.942			
CS2	0.936			
CS3	0.938			
**Entertainment services**		0.925	0.953	0.870
ES1	0.912			
ES2	0.908			
ES3	0.977			
**Social environment**		0.895	0.935	0.829
SE1	0.879			
SE2	0.975			
SE3	0.874			
**Physical appearance**		0.881	0.918	0.737
PHA1	0.821			
PHA2	0.878			
PHA3	0.876			
PHA4	0.856			
**Place image**		0.941	0.949	0.588
Entertainment services	0.815			
Social environment	0.835			
Physical appearance	0.871			
Community services	0.858			
**Pro-tourism behaviours**		0.921	0.944	0.808
PBI1	0.898			
PBI2	0.960			
PBI3	0.853			
PBI4	0.881			
**Chinese traditionality**		0.882	0.913	0.679
CT1	0.778			
CT2	0.913			
CT3	0.801			
CT4	0.725			
CT5	0.887			

*CR, composite reliability; AVE, average variance extracted*.

Fornell–Larcker criterion analysis and heterotrait–monotrait ratio of correlations (HTMT) are used to check discriminant validity. As shown in Table 3, all the square roots of each AVE value (in bold) are greater than their respective correlations across variables (Fornell and Larcker, 1981). Moreover, HTMT ratios (above the diagonal) were all less than the threshold of 0.9 (Henseler et al., 2015). Thus, the results confirm adequate discriminant validity.

**Table 3:** Correlations, AVE values, and HTMT ratios.

	**ATT**	**ATTT**	**PBI**	**CS**	**CT**	**ES**	**HTI**	**PHA**	**SE**
ATT	**0.897**	0.747	0.673	0.574	0.027	0.529	0.699	0.696	0.584
ATTT	0.696	**0.917**	0.610	0.684	0.063	0.609	0.795	0.736	0.599
PBI	0.627	0.577	**0.899**	0.470	0.092	0.429	0.623	0.505	0.524
CS	0.535	0.640	0.443	**0.939**	0.045	0.664	0.628	0.728	0.676
CT	−0.016	−0.062	−0.092	−0.038	**0.824**	0.035	0.030	0.066	0.024
ES	0.492	0.570	0.399	0.617	−0.015	**0.933**	0.647	0.641	0.642
HTI	0.648	0.745	0.582	0.585	−0.031	0.601	**0.937**	0.720	0.653
PHA	0.626	0.669	0.458	0.663	−0.051	0.586	0.654	**0.858**	0.724
SE	0.532	0.553	0.480	0.620	−0.012	0.588	0.598	0.645	**0.910**

*The square root of AVE is shown on the diagonal. Correlations across variables are below the diagonal, while HTMT ratios are above the diagonal*.

The article "How Residents' Attitudes to Tourists and Tourism Affect Their Pro-tourism Behaviours: The Moderating Role of Chinese Traditionality" was retracted in 2025. Reasons: unreliable results or conclusions; a conflict of interest; concerns about the peer review; concerns about the citations.

### Structural Model

Collinearity must be examined before the stage of the structural model. In this study, the variance inflation factor (VIF) values are used to check the tolerance of each variable. None of the VIFs exceed 5 (1–3.043) as a rule of thumb, suggesting that multicollinearity is not a limit in this study.

In the structural model step, coefficient of determination (*R*^2^), predictive relevance (*Q*^2^), statistical significance and relevance of the path coefficients were chosen for assessment. The *R*^2^-values in this study (ATT: 0.544; ATTT: 0.626; PBI: 0.479) are satisfactory. The *Q*^2^-values (ATT: 0.432; ATTT: 0.520; PBI: 0.370) also all have medium predictive relevance (Hair et al., 2019).

To evaluate the statistical significance and the relevance of the path coefficients in this study, a resampling method (5,000 samples) was used. As demonstrated in Table 4, residents' ATT was found to affect their PBI positively and significantly, thereby supporting H1. Residents' ATTT was found to influence their ATT positively and significantly, as predicted by H3. Residents' HTI significantly affected their ATT, ATTT and PBI, thus supporting H4, H5, and H6, respectively. Furthermore, residents' PI was found to be positively and significantly related to their ATTT and ATT, as predicted by H7 and H8, respectively. However, residents' ATTT and PI were found to have no significant influence on their PBI, so H2 and H9 were rejected.

**Table 4:** Results of hypotheses testing.

**Hypotheses**	**Path**	**Original sample**	**Standard error**	***t*-values**	***p*-values**	**Support**
H1	ATT → PBI	0.366	0.066	5.580	0.000	YES
H2	ATTT → PBI	0.134	0.088	1.529	0.126	NO
H3	ATTT → ATT	0.380	0.063	6.003	0.000	YES
H3a	ATTT → ATT → PBI	0.139	0.035	4.024	0.000	YES
H4	HTI → ATT	0.196	0.077	2.563	0.010	YES
H5	HTI → ATTT	0.465	0.061	7.679	0.000	YES
H6	HTI → PBI	0.218	0.070	3.130	0.002	YES
H6a	HTI → ATT → PBI	0.072	0.029	2.475	0.013	YES
H7	PI → ATTT	0.387	0.055	7.062	0.000	YES
H8	PI → ATT	0.234	0.075	3.116	0.002	YES
H9	PI → PBI	0.011	0.073	0.153	0.878	NO
H9a	PI → ATT → PBI	0.086	0.034	2.537	0.011	YES
H10	CT*ATT → PBI	0.176	0.066	2.668	0.008	YES
H11	CT*ATTT → PBI	−0.040	0.054	0.735	0.462	NO

All the hypothesised mediating effects of residents' ATT were found to be statistically significant (Table 4). As shown in Table 4, residents' ATTT, HTI and PI were all found to positively affect their PBI through ATT. H3a, H6a and H9a were all supported. The direct effect of residents' ATTT and PI on their PBI was not significant, confirming that residents' ATT fully mediated the relationships. The significant relationship between residents' HTI and PBI suggests that residents' ATT partially mediated the relationship.

The article "How Residents' Attitudes to Tourists and Tourism Affect Their Pro-tourism Behaviours: The Moderating Role of Chinese Traditionality" was retracted in 2025. Reasons: unreliable results or conclusions; a conflict of interest; concerns about the peer review; concerns about the citations.

The results also reveal that CT moderates the relationship between ATT and PBI, thereby supporting H10. However, the moderating effect of CT between ATTT and PBI was not significant, so H11 was rejected (Table 4; Figure 2).

**Figure 2:** Moderating effect of CT.

## Discussion and Conclusions

### Discussion

This study aims to further examine how HTI and PI influence residents' ATT and ATTT and ultimately their PBI by considering the moderating effect of CT into account and how their ATTT affect ATT. Of the 14 hypothesised relationships, 11 were supported. These findings contribute to the scholarly field of residents' PBI and shed light on the planning and management practises of places as tourist attractions for community planners and interested researchers.

The positive effect of residents' ATT on their PBI (supporting H1) reinforces previous studies' results (Chen and Raab, 2012; Moghavvemi et al., 2017; Ribeiro et al., 2017). Moghavvemi et al. (2017) found that residents' ATT has a significant effect on their support for tourism development. Ribeiro et al. (2017) also found a positive relationship between residents' positive attitudes and pro-tourism behaviour and a negative relationship between negative attitudes and pro-tourism behaviour. Chen and Raab (2012) drew a similar conclusion that residents' attitudes to community tourism were a valid predictor of their supportive intention. This positive relationship between attitudes and behaviours could also be further confirmed in certain theories, such as theory of reasoned action and social exchange theory (Shen et al., 2019), proving that attitude is an essential prerequisite of behaviour.

Regarding the influence of residents' ATTT on their ATT (supporting H3), the result obtained is in line with those of Woosnam (2012) and Hasani et al. (2016). Woosnam (2012) also found that welcoming nature and sympathetic understanding significantly. Hasani et al. (2016) found that welcoming nature, as one of the three dimensions of emotional solidarity which measure residents' ATTT, is the strongest factor affecting residents' attitudes to supporting tourism development. These consistent findings indicate that residents with positive ATTT are apt to hold positive ATT.

The article "How Residents' Attitudes to Tourists and Tourism Affect Their Pro-tourism Behaviours: The Moderating Role of Chinese Traditionality" was retracted in 2025. Reasons: unreliable results or conclusions; a conflict of interest; concerns about the peer review; concerns about the citations.

Residents' HTI positively influenced their ATT, ATTT and PBI (respectively confirming H4, H5, and H6), in line with previous studies. Eusébio et al. (2018) confirmed that HTI acts as the strongest determinant of residents' ATT. Joo et al. (2018) also found that the frequency and nature of residents' interactions with tourists can partially influence their emotional solidarity, a measure of residents' ATTT. Luo et al. (2015) drew a similar conclusion that contact between hosts and backpackers deepens hosts' understanding of backpackers and helps them evaluate backpackers' effects positively. These findings demonstrate that the more positive contact with tourists residents have, the more positive the stance they take towards tourists.

To the best of our knowledge, this study is one of the first attempts to test the direct influence of residents' PI on their ATTT (confirming H7). Our finding suggests a positive link between PI and ATTT, demonstrating that residents with favourable PI exhibit more positive ATTT than those with less favourable PI.

Referring to the relationship between residents' PI and ATT (supporting H8), results are consistent with those by Stylidis et al. (2014) and Stylidis et al. (2018). In Kavala, Stylidis et al. (2018) found that identified image-based residents shared dissimilar ATT. In the same city, residents' PI positively influences their level of support for tourism (Stylidis et al., 2014). In summation, these findings confirm that residents with more favourable PI tend to hold more positive ATT.

However, in contrast with some previous studies (Palmer et al., 2013; Martín et al., 2018), the positive effect of residents' ATTT on their PBI (predicted by H2) was not statistically significant. With a sample of 307 Welsh residents, Palmer et al. (2013) confirmed that residents' affective ATTT are related to their propensity to engage in positive advocacy to support inward tourism. In Santander and Torrelavega (Spain), Martín et al. (2018) found that local residents' ATTT positively influences residents' behaviour supporting tourism in host communities. The difference may be attributed to the differences between study areas and participants. Sirakaya et al. (2002) argued that factors that influence residents' support are likely to be dissimilar between developed and developing countries. Palmer et al. (2013) selected Wales, a developed country, as a study area, whereas we selected Huangshan City in China, a developing country. Moreover, an online survey was used to distribute questionnaires across the whole country in the study conducted by Palmer et al. (2013), while a face-to-face questionnaire was used in this study. In the study by Martín et al. (2018), the survey sites are the top two cities in the region of Cantabria, while Huangshan is a relatively small hinterland city. Huangshan City is the birthplace of Huizhou culture, which commonly holds having friends coming from distant quarters is a delightful notion. However, the local people are also very traditional and conservative. These phenomena may explain the different results between this study and those of Palmer et al. (2013), Martín et al. (2018).

The article "How Residents' Attitudes to Tourists and Tourism Affect Their Pro-tourism Behaviours: The Moderating Role of Chinese Traditionality" was retracted in 2025. Reasons: unreliable results or conclusions; a conflict of interest; concerns about the peer review; concerns about the citations.

Moreover, H9, which proposes that residents' BI depends on their PI, could not be confirmed, contradicting the findings of previous studies. In Eilat (Israel), Stylidis et al. (2017) found that the overall image of Eilat positively influenced local residents' intention to recommend the city to others. However, whereas these researchers used a single-item scale to measure PI and intention to recommend. Our measurement was more comprehensive, encompassing the four dimensions of CS, ES, SE and PHA. In another study on Eilat, Stylidis (2018) also found that three resident groups with different images of the city exhibited dissimilar intentions/behaviour towards tourism. The difference may be attributable to differences between the measurement of PI and participants. Stylidis (2018) used five types of attributes to measure PI (amenities, natural environment, SE, attractions, and accessibility), ignoring community attributes of the place for residents. By contrast, we used four types of attributes which consider destination and community attributes simultaneously to measure PI. The participants in this study consisted of not only permanent residents but also some immigrants in the area, whereas Stylidis (2018) only studied permanent residents. This lack of a link between residents' PI and their PBI in our study suggests the necessity of modifying the traditional approach of models aiming to understand the antecedents of residents' PBI.

In terms of the mediating effects of residents' ATT, to the best of our knowledge, our study is among one of the first in travel and tourism to test whether residents' ATTT, HTI and PI indirectly and positively affected their PBI through ATT. PI or ATTT would not have any influence on PBI without ATT, further demonstrating that ATT acts as the strongest predictor of PBI in this study. The partial mediation of ATT between HTI and PBI also demonstrates that residents' ATT strengthened the effect of their HTI on PBI.

As an individual cultural value, CT captures the core of Confucian ideology and Chinese culture. In this study, CT moderates the links between ATT and PBI (H10), meaning that the higher the residents CT, the stronger the influence of ATT on PBI. However, this scenario does not apply to the influences of ATTT (H11) because residents with a higher or lower level of CT do not demonstrate a significant difference in the conditional effect of ATTT on PBI. These findings contradict the statement of Azjen (1980) that the effect of individual attitudes on their intention formation may be determined by their value priorities. A possible major explanation for these disparities in findings is the insignificant relationship between ATTT and PBI in this study. Another explanation might be the different objects of attitudes, demonstrating the complexity of CT in moderating the links between attitudes and behaviour intention.

The article "How Residents' Attitudes to Tourists and Tourism Affect Their Pro-tourism Behaviours: The Moderating Role of Chinese Traditionality" was retracted in 2025. Reasons: unreliable results or conclusions; a conflict of interest; concerns about the peer review; concerns about the citations.

### Conclusions

This study investigates the role of HTI and PI in relation to ATT, ATTT and PBI using data from 357 residents living in Huangshan, a fifth-tier city in China. Some conclusions can be drawn from the findings. Firstly, ATT are the strongest predictor of PBI among all the independent variables (β = 0.366, *P* < 0.001), which is in line with most previous studies and some theories (e.g., theory of planned behaviour, theory of value–attitude–behaviour, attitude–behaviour–condition theory). Secondly, host–guest interaction demonstrates the most extensive impact on other variables, namely ATT, ATTT and PBI. Thirdly, as the strongest predictor, ATT mediates PI's, HTI's, and ATTTs' respective relationships with PBI. Lastly, the higher the CT of residents, the stronger the influence of their ATT on PBI.

## Theoretical and Practical Implications

This study investigates the effect of residents' HTI and PI on their ATT and ATTT and consequent reactions by considering the moderating effect of CT into account, contributing to the literature in the settings of travel and tourism. First, in accordance with the hypotheses, our findings revealed that residents' ATT significantly influenced their PBI. ATT was found to be the strongest predictor of residents' PBI in this study (β = 0.366, *P* < 0.001). These findings further consolidate the positive relationship between residents' ATT and their PBI in the related studies.

Second, this study introduced two types of residents' attitudes based on different objects (i.e., ATT and ATTT) into the research model simultaneously, bridging the gap in the previous literature that mainly focused on ATT as a predictor for PBI. The inconstant effects of attitudes on PBI also indicate that the objects of attitudes are crucial to the relationship between attitudes and consequent behaviours. The influence of residents' ATTT on their ATT is significant, suggesting a complex impact mechanism between differentiated types of resident attitudes and pointing the way forward for future research.

The article "How Residents' Attitudes to Tourists and Tourism Affect Their Pro-tourism Behaviours: The Moderating Role of Chinese Traditionality" was retracted in 2025. Reasons: unreliable results or conclusions; a conflict of interest; concerns about the peer review; concerns about the citations.

Third, residents' HTI positively influenced their ATT, ATTT and PBI, suggesting suggests that HTI may play a key role in shaping residents' ATT, ATTT, and PBI. These findings are in accordance with the call for in-depth examinations of intimacy and authenticity in how residents and tourists interact (Trauer and Ryan, 2005) and extend the limited existing literature on HTI from a resident perspective as a positive predictor of residents' ATT, ATTT, and PBI. Conversely, the effects of residents' PI and ATTT on their PBI have not been proven to be significant, suggesting the necessity of further examining these relationships in different settings. Notably, this study is the first to examine the effect of residents' PI on their ATTT. Future research is suggested to further verify this relationship.

Finally, this study is one of the first to explore the role of CT as a cultural boundary condition in the attitude–behaviour processes, particularly in non-western contexts such as Confucian China. This study empirically verified the statement of Azjen (1980) that the effect of individual attitudes on their intention formation may be determined by their value priorities. This finding contributes to academic considerations of the individual cultural value that could amplify or decrease influences of attitudes on intention, directing future research on the cultural boundary condition in the attitude–behaviour processes.

Our results also provide planners and practitioners with some valuable managerial advice to guide the improvement of tourist destinations. Owing to the positive influence of ATT on PBI, planners and practitioners should allow local communities to benefit more from tourism development, such as increased participation in the decision-making process, additional job opportunities and higher income. Tourism companies can also implement charity activities to form good reputations, significantly improving residents' attitudes towards tourism. Eventually, tourism companies will earn residents' support. Given that residents' HTI serves as an important determinant of their ATT, ATTT and PBI, community planners and practitioners are recommended to make policies that stimulate satisfactory interactions between residents and tourists. For instance, incentives should be given to residents if they carry out some local events and activities together with tourists (e.g., performing traditional dances, making handicrafts and preparing traditional meals). Some online resident and tourist group photo shows can also be organised. Tourists and residents in the selected group photo are rewarded, respectively. Tourists will receive travel packages and coupons, and residents are awarded the title of destination ambassador, and residents are awarded the title of destination ambassador. Although residents' PI cannot influence their PBI directly, it indirectly affects residents' PBI *via* ATT. Thus, policymakers and destination managers need to focus on improving residents' PI to gain their support. Concretely, potentially valuable initiatives include increasing job opportunities, protecting historic buildings, improving social security governance and increasing investment in infrastructure to enhance PI for local residents. Owing to the positive moderating effect of CT, integrating CT within tourist attractions development to gain residents' support is crucial. Specifically, local community planners and practitioners should strengthen the publicity of traditional culture, such as promoting Chinese figures in history, organising traditional cultural knowledge contests and producing excellent historical film shows and broadcasting. More historical and cultural museums should be open to the public for free and the proportion of traditional cultural education in the curriculum should be increased in schools. Planners and practitioners should also place a high value on and pay attention to the concerns of respectable male seniors to gain their support. For instance, free medical examinations and birthday gifts should be offered every year for the elderly in the surrounding communities of attractions.

The article "How Residents' Attitudes to Tourists and Tourism Affect Their Pro-tourism Behaviours: The Moderating Role of Chinese Traditionality" was retracted in 2025. Reasons: unreliable results or conclusions; a conflict of interest; concerns about the peer review; concerns about the citations.

In sum, this study will benefit planners and practitioners in deepening their understanding of the complexity of factors that can affect residents' PBI, which is especially important to maintain the sustainability of other cities similar to Huangshan.

## Limitations and Future Research

Despite the contributions of this study, several limitations should be noted. First, because the questionnaires were distributed and gathered in the surrounding communities of Huangshan Scenic Area, residents from inner-city locations were excluded. Thus, the significance and strength of the relationships may be differential. Another limitation is that Huangshan City, as the birthplace of Huizhou culture, is a relatively small hinterland city, and local people might be more traditional and conservative than those from big cities. Therefore, future research could select places with different cultural backgrounds to examine whether the same results will be obtained. Last but not least, this study was conducted during the COVID-19 pandemic, and future research might investigate whether and how COVID-19 affects these behaviours.

The article "How Residents' Attitudes to Tourists and Tourism Affect Their Pro-tourism Behaviours: The Moderating Role of Chinese Traditionality" was retracted in 2025. Reasons: unreliable results or conclusions; a conflict of interest; concerns about the peer review; concerns about the citations.

## Data Availability Statement

The raw data supporting the conclusions of this article will be made available by the authors, without undue reservation.

## Author Contributions

KS and JY conceived the study. KS, JY, and CG wrote the manuscript. All authors designed the study, collected and analysed the data, read and approved the manuscript, and agreed to be accountable for all aspects of the work.

## Funding

This research was funded by Anhui Province Higher Education Humanities and Social Science Research Project (SK2020A0465) and Huangshan University Research Foundation for Talented Scholars (2020xskq005).

## Conflict of Interest

The authors declare that the research was conducted in the absence of any commercial or financial relationships that could be construed as a potential conflict of interest.

## Publisher's Note

All claims expressed in this article are solely those of the authors and do not necessarily represent those of their affiliated organizations, or those of the publisher, the editors and the reviewers. Any product that may be evaluated in this article, or claim that may be made by its manufacturer, is not guaranteed or endorsed by the publisher.

## Footnotes

^1^http://tjj.ah.gov.cn/ssah/qwfbjd/tjgb/sjtjgbao/118163911.html.
